# Serum Pharmacochemistry Analysis Using UPLC-Q-TOF/MS after Oral Administration to Rats of Shenfu Decoction

**DOI:** 10.1155/2015/973930

**Published:** 2015-07-27

**Authors:** Jia-le He, Jia-wei Zhao, Zeng-chun Ma, Yu-guang Wang, Qian-de Liang, Hong-ling Tan, Cheng-rong Xiao, Xiang-lin Tang, Yue Gao

**Affiliations:** ^1^Graduate School, Anhui Medical University, Hefei, China; ^2^Beijing Institute of Radiation Medicine, Tai-Ping Road 27, Beijing 100850, China

## Abstract

The purpose of this study was to study the serum pharmacochemistry of SFD as well as the material basis through analyzing the constituents absorbed in blood. The SFD was orally administrated to Wistar rats at 20 g·kg^−1^, and Ultra Performance Liquid Chromatography (UPLC) fingerprints of SFD were created. Serum samples were collected for analysis, and further data processing used MarkerLynx XS software. 19 ginsenosides and 16 alkaloids were detected in SFD. The absorption of alkaloids (mainly monoester diterpenoid alkaloids) increased when* Aconitum carmichaeli* Debx. was combined with* Panax ginseng*, while the ginsenosides remained stable. Diester diterpenoid alkaloids were not present in the serum samples. A suitable serum pharmacochemistry method was successfully established to study pharmacological effects and potential improvements in formulation. This may also be useful for toxicity reduction. We suspect that the increased absorption of the monoester diterpenoid alkaloids from the mixture of* Panax* and* Radix*, compared to the* Panax* only extract, may be the reason for the combination of the two herbs in popular medicine formulas in China.

## 1. Introduction

Shenfu Decoction (SFD) consisting of an equal ratio of ginseng root (radix ginseng, Renshen) and aconite root (*Radix Aconiti Lateralis Preparata*, Fuzi) is an example of a classic Chinese traditional herb-couple formulation, where two herbs are prescribed together to decrease toxicity and/or increase efficacy. For example, inclusion of* Glycyrrhiza uralensis* can prevent or destroy the toxicity of treated Fuzi [1]. The main components are ginsenosides and alkaloids. SFD was originally described in* Ji Sheng Xu Fang* (1253 in western calendar) written by Yonghe in the Song Dynasty. In many formulae of Traditional Chinese Medicine (TCM), Renshen is frequently prescribed in combination with other herbs to decrease toxicity and increase efficacy. Ginsenosides are the main bioactive constituents in the famous Chinese herb Renshen. They include protopanaxadiol, protopanaxatriol, octotillol, and oleanolic acid. Aconitines are the main constituents in* Aconitum carmichaelii* Debx. Aconitines include monoester diterpenoid alkaloids (MDAs) and diester diterpenoid alkaloids (DDAs) and have differences in esterification. Their chemical structures are shown in Figure 1. Due to the high toxicity of DDAs,* Fuzi* is combined with* Renshen* to decrease its toxicity.

SFD is used to treat cardiovascular diseases such as circulatory collapse, shock, thoracic obstruction, and acute thoracic pain. It has a therapeutic effect on heart failure and ischemia-reperfusion injury [2]. One study showed that blockage of the sodium channels in cardiac myocytes may be one of the important molecular mechanisms of its cardiac effect [3]. There are no detailed studies of its mechanism of action, and the bioactive compounds that account for its therapeutic effects remain unclear.

While they have the so-called active ingredients, there are no empirical data to prove its effectiveness. Oral administration is one of the primary modes for TCM. The bioactive compounds are absorbed in the blood and transferred to the target. Thus, while there are multiple components in herbs, only those that are absorbed into circulation are effective [4].

Pharmacokinetics remains unresolved in the use of Chinese herbs. In our previous research, we focused on the influence of DDAs, drug metabolism enzymes, and transporters after the combination of* Renshen* and* Fuzi* [5–7]. Our previous study* in vitro* showed that there were significant differences between codecoction and mixed decoction of* Renshen* and* Fuzi* [5]. The content of toxic alkaloids was higher in mixed decoction than codecoction which was probably the attenuation basis. To confirm whether they behaved similarly* in vivo* is one of our goals. Here, we developed a rapid and sensitive Ultra Performance Liquid Chromatography/Quadrupole Time-of-Flight Mass Spectrometry (UPLC/Q-TOF-MS) method to study the pharmacokinetics of SFD constituents.

## 2. Materials and Methods

### 2.1. Chemicals and Materials

HPLC-grade acetonitrile was purchased from Fisher Scientific (Waltham, MA, USA). Methanol was purchased from Sinopharm Chemical Reagent Co. (Shanghai, China). Formic acid was HPLC-grade (CNW Technologies GmbH, Dusseldorf, Germany). Renshen and Fuzi were purchased from Hebei Anguo Drug Market (Hebei, China) and authenticated by Professor Baipin Ma, Institute of Radiation Medicine Sciences of the Academy of Military Medical Sciences. The Renshen was at least 5-year growth white ginseng which was processed by the method of the* Chinese Pharmacopoeia* (2010) and the Fuzi was nonprocessed* Radix Aconiti Lateralis Preparata* (only for laboratory use). The vouched specimens were stored in storage room of the Department of Pharmacology and Toxicology of the Institute of Radiation Medicine Sciences of the Academy of Military Medical Sciences.

### 2.2. Preparation of Decoction and for LC-MS Analysis

Renshen (100 g) was soaked in 800 mL distilled water for 30 min and decocted for 1 h and then filtered. The residue was decocted in 500 mL distilled water for 1 h and filtered. The filtrate was then combined and labeled Renshen decoction. Fuzi (100 g) was decocted in 800 mL distilled water for 10 min and then filtered. The residue was decocted in 500 mL distilled water for 30 min and filtered and labeled Fuzi decoction. Then two different kinds of decoctions were prepared, namely, Renshen-Fuzi codecoction where the two herbs mixed together were extracted with water and Renshen-Fuzi mixed decoction where the individual herbs were extracted separately with water and the extracts then mixed together. The decoctions were evaporated to 1 g crude herb per mL. The decoctions were stored at 4°C, and the decoction samples were subjected to UPLC/Q-TOF-MS analysis, and the datasets were processed with MassLynx software.

### 2.3. Animals Handling and Serum Samples Preparation

Forty male Wistar rats (200 ± 20 g) were obtained from the Laboratory Animal Center of the Academy of Military Medical Sciences (Beijing, China, production certificate number SCXK-(M) 2007-004). All procedures were performed in accordance with the protocol outlined in the* Guide for the Care and Use of Laboratory Animals* published by the US National Institute of Health (NIH publication number 85-23, revised 1996) and approved by the Committee on the Ethics of Animal Experiments of the Academy of Military Medical Sciences. They were randomly divided into 5 groups: blank group (B-Group),* Renshen* decoction group (R-Group),* Fuzi* decoction group (F-Group), codecoction group (C-Group), and mixed decoction group (M-Group). There were 8 rats in each group. The rats were kept in an animal room with controlled environment (temperature: 22 ± 2°C, relative humidity: 55 ± 5%, and 12 h light-dark cycle) for 3 days before the experiment. All animals were free to access distilled water and standard food.

Every group except the blank group received an oral administration of 20 g·kg^−1^ decoction for 3 days. A distilled water vehicle control was given to the blank group. Blood samples (500 *μ*L) were collected from the retroorbital sinus 1 h after oral administration on the 3rd day and centrifuged at 3000 rpm for 10 min. Then, 800 *μ*L methanol was added to the 200 *μ*L serum samples, vortexed, and then centrifuged at 13000 rpm for 10 min. The supernatant solution was transferred to another tube and dried with nitrogen gas. The residue was stored in 50% acetonitrile (200 *μ*L) and frozen at −80°C until analysis.

### 2.4. Instrumentation and Chromatographic Conditions

#### 2.4.1. Ultra Performance Liquid Chromatography

Chromatographic analysis was performed with an ACQUITY Ultra Performance Liquid Chromatography system (Waters, USA) controlled with MassLynx V4.1 software. Separation used an ACQUITY UPLC HSS T3 Column (2.1 × 100 mm, 1.8 *μ*m, Waters). Water with 0.1% formic acid (v/v) and acetonitrile with 0.1% formic acid (v/v) were used as mobile phases A and B, respectively, at a flow rate of 0.45 mL·min^−1^. The gradient conditions of the mobile phase in positive mode were 0–2 min: 5% B; 2–6 min: 5–12% B; 6–8 min: 12–20% B; 8–16 min: 20–50% B; 16-17 min: 50–5% B; and 17-18 min: 5% B. The gradient conditions of the mobile phase in negative mode were 0-1 min: 25% B; 1–3 min: 25–30% B; 3–16 min: 30–35% B; 16-17 min: 35-25% B; and 17-18 min: 25% B.

#### 2.4.2. Mass Spectrometry

A Waters Synapt High-Definition Time-of-Flight Mass Spectrometry (TOF-MS) system (Waters) equipped with an electrospray ionization (ESI) source operating in positive and negative mode was connected to the UPLC. A capillary voltage of 2.9 and 3.0 kV was used in positive and negative ionization mode, respectively. The desolvation temperature was 450°C, and the sampling cone voltage was 40 V. The extraction cone voltage was 4.0 V, source temperature was 100°C, and cone gas flow was 50 L·h^−1^. The desolvation gas flow rate was 900 L·h^−1^ in both positive and negative ionization modes. The mass was corrected during acquisition with leucine-enkephalin to generate a reference ion at* m/z *556.2771 Da ([M + H]^+^) in positive ion mode and* m/z *554.2615 Da ([M − H]^−^) in the negative ion mode. This ensured accurate mass measurements.

### 2.5. Data Analysis

All data were processed by MassLynx V4.1 software (Waters). The chromatographic peaks were integrated, aligned, and combined with accurate mass to charge ratios. A reference retention time was found for each expected compound. Using our previous work, the compounds in the decoction were identified [8–10]. The data were further processed by MarkerLynx XS software (Waters). The exported data list, partial least-squares-discriminant analysis (PLS-DA) as well as principal component analysis (PCA), was used to analyze the differences between the groups.

## 3. Results

### 3.1. Chemical Analysis of Codecoction

The ginsenosides and alkaloids in SFD were identified using UPLC combined with a TOF-MS detector. The total ion chromatogram of SFD in positive and negative ion modes is shown in Figure 2 and was processed with MassLynx V4.1 (Waters, USA). Comparing the retention time and mass data with reference compounds identified the target compounds. Both the MDAs and DDAs of alkaloids and 20(s)-protopanaxadiol type, 20(s)-protopanaxatriol type, and oleanolic acid saponin-type ginsenosides were detected in SFD. The chemical compositions are shown in Tables 1 and 2.

### 3.2. Alkaloids Difference in Serum Detected by Positive Mode

#### 3.2.1. Differences in the Five Groups

All five groups were processed by PLS-DA and were used to highlight variation among the five groups (see Figure 3). Exported PCA plots and loading plots showed that the five groups formed five clusters. This indicated that the components in the serum were different.

#### 3.2.2. Alkaloids Difference between B-Group, F-Group, M-Group, and C-Group

Comparing F-Group with B-Group, 14 kinds of alkaloids including DDAs, MDAs, and general alkaloids in aconitum plants were detected. Most of them were trace amount, which indicated the alkaloids poor absorption* in vivo*. The main reason was high efflux ratio reduced by P-glycoprotein [11–13]. These 14 kinds of alkaloids might be the chemical constituents involved in therapeutic efficacy of SFD. Some researchers thought that Fuzi's therapeutic activity (anti-inflammatory, analgesic, and cardiotonic activity) seems to have relevance to the presence of toxic alkaloids [14, 15] but the other researchers thought that Fuzi's toxicity compounds (mainly aconitine, mesaconitine, and hypaconitine) are not essential for its efficacy [16] (see Figure 4).

After detecting these 14 alkaloids, we further processed the data. Comparing C-Group with F-Group, the absorption of MDAs (benzoylaconine, mesaconine, 10-OH-benzoylmesaconine, and dehydrated benzoylmesaconine) decreased and the general alkaloids in aconitum plants (cammaconine, neoline, and talatizamine) increased. Most alkaloids (cammaconine, carmichaeline, talatizamine, acetyltalatizamine, and dehydrated benzoylhypaconine) absorption in M-Group was increased rather than F-Group. The increased or decreased absorption of alkaloids may contribute to the attenuation and synergistic effects. The decreased absorption of toxic alkaloids leads to attenuation and increased nontoxic alkaloids contribute to synergistic effects mainly because of compatibility of Renshen. The phenomenon was found in ancient year by the Chinese and we make it clear by analyzing the chemical compounds (see Figures 5 and 6).

The M-Group data showed that all alkaloids were absorbed more than the C-Group. The relative intensity of the ion indicated that the toxic chemicals (mesaconine, 10-OH-benzoylmesaconine, dehydrated benzoylmesaconine, and dehydrated benzoylhypaconine) were less absorbed than most general alkaloids in* Aconitum* plants (cammaconine, carmichaeline, fuziline, talatizamine, acetyltalatizamine, and neoline). The content of toxic alkaloids was higher in mixed decoction than codecoction which was probably the attenuation basis* in vitro*, and the results* in vivo* showed a similar consequence which indicated that the* Renshen* attenuated the toxicity of* Fuzi*. And ester exchange or degradation reactions occurring during the processing of codecoction with Renshen were considered to be the key factor of attenuation [5] (see Figure 7).

#### 3.2.3. Ginsenosides Differences in the Serum in Negative Mode

The ginsenosides and alkaloids were detected in negative and positive mode, respectively. In our study, the codecoction and mixed decoction had small differences in the negative mode. This indicated that the ginsenosides behaved similarly, and the results presented the same tendency with an unpublished paper for the negative result* in vitro*. The same processing method used in positive mode was also applied to negative mode to analyze the ginsenoside differences. The PCA and PLS-DA/S-Plot showed no obvious distinction between the C-Group and the M-Group. However, 13 kinds of ginsenosides (GRg_1_, GRe, GRd, GRo, GRc, GRb_2_, GRb_3_, GRb_1_, GRa_2_, GRa_1_, MalonylGRc, MalonylGRb_1_, and MalonylGRb_2_) were detected in the serum of the* Panax ginseng* group. The extracted ion chromatogram and mass spectrogram of the ginsenosides are shown in Figures 8, 9, and 10.

## 4. Discussion

Researchers have reported quantitative analysis of aconitum alkaloids of SFD* in vitro* as well as the pharmacokinetic behavior of* Fuzi* and drug-drug interaction mechanisms in herb pair decoctions [17–19]. Relatively few studies have been conducted on the material basis of SFD* in vivo*, and most researchers focused on Shenfu injection which is a kind of processed Shenfu formulation [20, 21]. The material basis of toxicity reduction and pharmacological effect improvement* in vivo* remains unclear. In previous studies, the attenuation and synergistic effects of SFD including decoction time and herb ratio were studied* in vitro*. However, aconitum alkaloids serum levels were difficult to detect after oral administration, and only trace level was seen for its low bioavailability [18, 22]. Only Shenfu injected powder showed detectable alkaloids in serum [23]. Multicomponents and multitarget herbs resulted in complex systems with difficult detection. Recently, UPLC coupled with TOF-MS has become a vitally important tool in studying Chinese herbs. It is fast with good selectivity, high resolution, and accurate mass measurements. This makes it attractive for the analysis of complex biological sample [24].

Shenfu formulation was a classical Chinese medicine for its obvious therapy efficiency on heart fail [25], but* Fuzi* in the formulation was a famous toxicity herb for its severe arrhythmia and neurological, cardiovascular, and gastrointestinal symptoms [26]. The herb pair was used for synergism and attenuation and the decoction method was thought to be the main reason for its chemical difference, but whether it behaves similarly* in vivo* was still a mystery, and here we approved an evidence to evaluate the Shenfu formulation* in vivo*. The concentration of hypaconitine and deoxyaconitine decreased, while benzoylmesaconine, benzoylhypaconine, and dehydrated benzoylmesaconine increased in the codecoction samples. The toxicity increased in single decocted or mixed decocted samples [5]. The codecoction inhibited toxic compounds, and the inhibited alkaloids dissolution resulted in a lower alkaloids content in the C-Group than the M-Group. They behaved similarly* in vivo* and* in vitro*. Here,* Renshen* showed evidence of increasing the absorption of alkaloids. These alkaloids were measured in a relative concentration range and found to be in accordance with the tradition of TCM. We suspect that toxicity reduction is due to decoction* in vitro*; the pharmacological effect improvement is due to increased absorption and metabolism* in vivo*.

The pharmacological effect* in vivo* was affected by absorption and metabolism. In previous study, alkaloids were metabolized by Cytochrome P450 (CYP450) 3A [27]. A study on Shenfu injection indicated that it inhibited the enzyme activity of CYP3A at the mRNA level [6]. Mean Residence Time (MRT) increased when the enzyme activity was inhibited. Its absorption increase contributed to an increase in the Area under the Curve (AUC). The increased MRT and AUC indicated an increase in pharmacological effects.

Efflux transporters in the intestine play an important role in absorption. They also protect the body from toxin damage. The ATP-binding cassette transporters include P-glycoprotein (P-gp), multidrug resistance-associated protein isoform 2 (MRP2), and breast cancer resistance protein (BCRP). They modulate the absorption, distribution, metabolism, and excretion of medicine. These proteins are highly expressed in the apical membranes of intestinal epithelial, hepatic, and renal tubular cells. Transport studies show that the efflux ratios of aconitine, mesaconitine, and hypaconitine were significantly elevated due to P-gp and BCRP [11].* Panax ginseng* and ginsenosides like ginsenoside F1, ginsenoside Re, and ginsenoside Rb_2_ induced the function of P-gp [28]. An important clue is seen in that Fuzi's toxicity compounds (aconitine, mesaconitine, and hypaconitine) are not essential for its efficacy [16]. While aconitine, mesaconitine, and hypaconitine were not detected in serum, it could be because they were below the detection limit.

The difference in molecular structure between DDAs and MDAs is an acetyl group. This caused the different efflux ratios. The lost acetyl group decreased the toxicity of the DDAs and the efflux ratio [29]. In another TCM herb pair* Fuzi-Ganjiang* formula,* Ganjiang* (*Rhizoma Zingiberis*, derived from the dry rhizome of* Zingiber officinale* Rosc.) was combined with* Fuzi* to decrease its toxicity and improve pharmacological effects. The authors showed that* Ganjiang* enhanced the absorption of MDAs and promoted the elimination of DDAs [30]. We could hypothesize that* Renshen* played the same role in these herb pairs. Our findings showed that nontoxic alkaloids in the M-Group and C-Group absorption increased more than F-Group. The absorption of alkaloids in mixtures or extractions was better than that of pure compounds seen in other experiments [12].

Like many other TCMs, SFD is always taken orally. Ginsenosides showed poor absorption and low bioavailability [31]. Major factors that limited the intestinal absorption of ginsenosides were poor membrane permeability and active biliary excretion. This limited systemic exposure to most ginsenosides and their deglycosylated metabolites [32]. The poor absorption and bioavailability of ginsenoside make them difficult to accurately measure in serum. Thus, we successfully developed a new method to measure ginsenoside previously. The different clearance rate of ginsenosides is considered to be the mechanism of Shenfu injection [10].

In the past decades, researchers have studied traditional Chinese formulas sufficiently, but the material basis and mechanism are still unclear with most data focusing on pharmacokinetics. Most studies are multicomponent herbs and with multiple targets* in vivo*. In addition to active compounds, there are also inactive and even toxic compounds in herbs. The material basis, pharmacology, component compatibility, and physiological disposition of TCM remain unclear. Understanding the attenuation and synergistic effects on absorption is an important goal of this study. Here, we studied the material basis of attenuation and synergistic effects by measuring the absorbed ingredients.

## Figures and Tables

**Figure 1:** The chemical structure of 20(S)- and 20(R)-protopanaxadiol ginsenosides (a), 20(S)- and 20(R)-protopanaxatriol ginsenosides (b), oleanolic acid saponins type (c), and aconitines (d).

**Figure 2:** Total ion chromatogram of codecoction. (a) Positive ion mode detected alkaloids, (b) negative ion mode detected ginsenosides.

**Figure 3:** (a) PLS-DA loadings plot of five groups. (b) PCA score plot of the five groups. B-Group: blank group; R-Group: Renshen decoction group; F-Group: Fuzi decoction group; C-Group: codecoction group; M-Group: mixed decoction group. There were 8 rats in each group and each received an oral administration of 20 g·kg^−1^ decoction for 3 days. The blank group received an equivalent volume of distilled water.

**Figure 4:** Relative content of alkaloids detected in F-Group serum. F-Group: Fuzi decoction group; A: cammaconine; B: carmichaeline; C: fuziline; D: neoline; E: talatizamine; F: acetyltalatizamine; G: mesaconine; H: 10-OH-benzoylmesaconine; K: benzoylaconine; M: benzoylmesaconine; N: dehydrated benzoylmesaconine; X: dehydrated benzoylhypaconine; Y: 10-OH-mesaconitine; Z: hypaconitine.

**Figure 5:** Relative content of alkaloids detected in rats serum of F-Group and C-Group. F-Group: Fuzi decoction group; C-Group: codecoction group. A: cammaconine; B: carmichaeline; C: fuziline; D: neoline; E: talatizamine; K: benzoylaconine; G: mesaconine; H: 10-OH-benzoylmesaconine; N: dehydrated benzoylmesaconine; X: dehydrated benzoylhypaconine.

**Figure 6:** Relative content of alkaloids detected in rats serum of F-Group and M-Group. F-Group: Fuzi decoction group; M-Group: mixed decoction group. A: cammaconine; B: carmichaeline; C: fuziline; D: neoline; E: talatizamine; F: acetyltalatizamine; K: benzoylaconine; G: mesaconine; H: 10-OH-benzoylmesaconine; M: benzoylmesaconine; N: dehydrated benzoylmesaconine; X: dehydrated benzoylhypaconine.

**Figure 7:** Relative content of alkaloids detected in rats serum of C-Group and M-Group. C-Group: codecoction group; M-Group: mixed decoction group. A: cammaconine; B: carmichaeline; C: fuziline; D: neoline; E: talatizamine; F: acetyltalatizamine; G: mesaconine; H: 10-OH-benzoylmesaconine; M: benzoylmesaconine; N: dehydrated benzoylmesaconine; X: dehydrated benzoylhypaconine.

**Figure 8:** (a) PCA scores plot of C-Group and M-Group. (b) PLS-DA loadings plot of five groups. B-Group: blank group; R-Group: Renshen decoction group; F-Group: Fuzi decoction group; C-Group: codecoction group; M-Group: mixed decoction group. There were 8 rats in each group and each received an oral administration of 20 g·kg^−1^ decoction for 3 days. The blank group received an equivalent volume of distilled water.

**Figure 9:** Extracted ion chromatogram of ginsenoside in negative ion mode. A_1_: GRg_1 _(Rt 2.40,* m/z *845.4856), B_1_: GRe (Rt 2.36,* m/z *991.5491), C_1_: GRd (Rt 14.72,* m/z *991.5526), D_1_: GRo (Rt 9.34,* m/z *955.4781), E_1_: GRc (Rt 10.09,* m/z *1077.5908), F_1_: GRb_2 _(Rt 11.49,* m/z *1077.5840), G_1_: GRb_3 _(Rt 11.97,* m/z *1077.5867), H_1_: GRb_1 _(Rt 8.78,* m/z *1107.6164), M_1_: MalonylGRc (Rt 10.56,* m/z *1163.5669), N_1_: MalonylGRb_1 _(Rt 12.35,* m/z *1163.5894), X_1_: MalonylGRb_2_ (Rt 9.53,* m/z *1193.5908), Y_1_: GRa_2_ (Rt 8.34,* m/z *1209.6553), Z_1_: GRa_1_ (Rt 8.37,* m/z *1209.6318).

**Figure 10:** Mass spectrogram of ginsenoside in negative ion mode. A_1_: GRg_1 _(Rt 2.40,* m/z *845.4856), B_1_: GRe (Rt 2.36,* m/z *991.5491), C_1_: GRd (Rt 14.72,* m/z *991.5526), D_1_: GRo (Rt 9.34,* m/z *955.4781), E_1_: GRc (Rt 10.09,* m/z *1077.5908), F_1_: GRb_2 _(Rt 11.49,* m/z *1077.5840), G_1_: GRb_3 _(Rt 11.97,* m/z *1077.5867), H_1_: GRb_1 _(Rt 8.78,* m/z *1107.6164), M_1_: MalonylGRc (Rt 10.56,* m/z *1163.5669), N_1_: MalonylGRb_1 _(Rt 12.35,* m/z *1163.5894), X_1_: MalonylGRb_2_ (Rt 9.53,* m/z *1193.5908), Y_1_: GRa_2_ (Rt 8.34,* m/z *1209.6553), Z_1_: GRa_1_ (Rt 8.37,* m/z *1209.6318).

**Table 1:** Alkaloids detected from codecoction.

Peak number	*t*_*R*_ (min)	Assigned identity	Molecular formula	[M + H]^+^/*m*/*z*		
				Mean measured mass (Da)	Theoretical exact mass (Da)	Mass difference (ppm)
1	4.19	Mesaconine	C_24_H_39_O_9_N	486.2725	486.2703	4.52
2	4.73	Carmichaeline	C_22_H_35_O_4_N	378.2661	378.2644	4.49
3	4.86	Cammaconine	C_23_H_37_O_5_N	408.2751	408.2750	0.24
4	6.39	Fuziline	C_24_H_39_O_7_N	454.2806	454.2805	0.22
5	6.93	Neoline	C_24_H_39_O_6_N	438.2863	438.2856	1.60
6	7.79	Talatizamine	C_24_H_39_O_5_N	422.2898	422.2906	−1.89
7	9.05	Acetyltalatizamine	C_26_H_41_O_6_N	464.3036	464.3012	5.17
8	9.16	10-OH-Benzoylmesaconine	C_31_H_43_O_11_N	606.2959	606.2914	7.42
9	10.36	Benzoylmesaconine	C_31_H_43_O_10_N	590.2980	590.2965	2.54
10	11.01	Benzoylaconine	C_32_H_45_O_10_N	604.3125	604.3122	0.50
11	11.10	Dehydrated benzoylmesaconine	C_31_H_41_O_9_N	572.2861	572.2860	0.17
12	11.86	10-OH-Mesaconitine	C_33_H_45_O_12_N	648.3018	648.3020	−0.31
13	12.36	Dehydrated benzoylhypaconine	C_31_H_41_O_8_N	556.2919	556.2910	1.62
14	12.70	Mesaconitine	C_33_H_45_O_11_N	632.3054	632.3071	−2.69
15	13.61	Hypaconitine	C_33_H_45_O_10_N	616.3087	616.3122	−5.68
16	14.58	Deoxyaconitine	C_34_H_47_O_10_N	630.3254	630.3278	−3.81

**Table 2:** Ginsenoside identified from codecoction.

Peak number	*t*_*R*_ (min)	Assigned identity	Molecular formula	[M − H]^−^ ([M – H + HCOOH]^−^)/*m*/*z*		
				Mean measured mass (Da)	Theoretical exact mass (Da)	Mass difference (ppm)
1	1.72	Notoginsenoside R_1_	C_47_H_80_O_18_	977.5322	977.5321	0.10
2	1.76	20-Glucosylginsenoside Rf	C_48_H_82_O_19_	961.5309	961.5372	−0.31
3	2.19	Ginsenoside Re	C_48_H_82_O_18_	991.5481	991.5478	0.30
4	2.23	Ginsenoside Rg_1_	C_42_H_72_O_14_	845.4880	845.4899	−2.25
5	5.23	Ginsenoside Rf	C_42_H_72_O_14_	799.4845	799.4844	0.13
6	6.06	Ginsenoside F_3_	C_41_H_70_O_13_	769.4738	769.4738	0.00
7	6.15	20(R)-Ginsenoside Rg_2_	C_42_H_72_O_13_	783.4873	783.4895	−2.81
8	7.01	Ginsenoside F_2_	C_42_H_72_O_13_	829.4943	829.4950	−0.84
9	7.69	Ginsenoside Ra_2_	C_58_H_98_O_26_	1209.5927	1209.5904	1.90
10	7.71	Ginsenoside Ra_1_	C_58_H_98_O_26_	1209.5928	1209.5904	1.98
11	8.11	Ginsenoside Rb_1_	C_54_H_92_O_23_	1107.5935	1107.5951	−1.44
12	8.70	Ginsenoside Ro	C_48_H_76_O_19_	955.4913	955.4903	1.05
13	8.78	Malonylginsenoside Rb_1_	C_57_H_94_O_26_	1193.6003	1193.5955	4.02
14	9.33	Ginsenoside Rc	C_53_H_90_O_22_	1077.5854	1077.5846	0.74
15	10.12	Malonylginsenoside Rc	C_56_H_92_O_25_	1163.5876	1163.5850	2.23
16	10.64	Ginsenoside Rb_2_	C_53_H_90_O_22_	1077.5871	1077.5846	2.32
17	11.12	Ginsenoside Rb_3_	C_53_H_90_O_22_	1077.5871	1077.5846	−0.56
18	11.45	Malonylginsenoside Rb_2_	C_56_H_92_O_25_	1163.5879	1163.5850	2.49
19	13.76	Ginsenoside Rd	C_48_H_82_O_18_	991.5476	991.5478	−0.20
20	15.25	Ginsenoside Ma-Rd	C_51_H_84_O_21_	1031.5454	1031.5427	2.62

## Abbreviations

AUC: Area under the Curve
B-Group: Blank group
BCRP: Breast cancer resistance protein
C-Group: Codecoction group
CYP450: Cytochrome P450
DDAs: Diester diterpenoid alkaloids
F-Group: Fuzi decoction group
MRT: Mean Residence Time
MDAs: Monoester diterpenoid alkaloids
M-Group: Mixed decoction group
MRP2: Multidrug resistance-associated protein isoform 2
P-gp: P-glycoprotein
PLS-DA: Partial least-squares-discriminant analysis
PCA: Principal component analysis
R-Group: Renshen decoction group
SFD: Shenfu Decoction
TCM: Traditional Chinese Medicine
UPLC/Q-TOF-MS: Ultra Performance Liquid Chromatography/Quadrupole Time-of-Flight Mass Spectrometry.
